# Skin Diseases Classification Using Hybrid AI Based Localization Approach

**DOI:** 10.1155/2022/6138490

**Published:** 2022-08-29

**Authors:** Keshetti Sreekala, N. Rajkumar, R. Sugumar, K. V. Daya Sagar, R. Shobarani, K. Parthiban Krishnamoorthy, A. K. Saini, H. Palivela, A. Yeshitla

**Affiliations:** ^1^Department of CSE, Mahatma Gandhi Institute of Technology, Hyderabad, Telangana, India; ^2^Department of CSE, Vel Tech Rangarajan Dr. Sagunthala R&D Institute of Science and Technology, Chennai, Tamilnadu, India; ^3^Department of Computer Science and Engineering, MITSOE, MITADT University, Pune, India; ^4^Department of Electronics and Computer Science, Koneru Lakshmaiah Education Foundation, Vaddeswaram, Guntur, Andhra Pradesh, India; ^5^Department of Computer Science and Engineering, Dr. M.G.R Educational and Research Institute, Maduravoyal, Chennai, Tamilnadu, India; ^6^School of Computer Science and Engineering, Vellore Institute of Technology, Vellore, Tamilnadu, India; ^7^Department of Computer Science and Engineering, GBPIET, Pauri Garhwal, Uttarakhand, India; ^8^Accenture Solutions, Mumbai, Maharashtra, India; ^9^Department of Biotechnology, College of Biological and Chemical Engineering, Addis Ababa Science and Technology University, Addis Ababa, Ethiopia

## Abstract

One of the most prevalent diseases that can be initially identified by visual inspection and further identified with the use of dermoscopic examination and other testing is skin cancer. Since eye observation provides the earliest opportunity for artificial intelligence to intercept various skin images, some skin lesion classification algorithms based on deep learning and annotated skin photos display improved outcomes. The researcher used a variety of strategies and methods to identify and stop diseases earlier. All of them yield positive results for identifying and categorizing diseases, but proper disease categorization is still lacking. Computer-aided diagnosis is one of the most crucial methods for more accurate disease detection, although it is rarely used in dermatology. For Feature Extraction, we introduced Spectral Centroid Magnitude (SCM). The given dataset is classified using an enhanced convolutional neural network; the first stage of preprocessing uses a median filter, and the final stage compares the accuracy results to the current method.

## 1. Introduction

There are a lot of hidden problems in the skin that may occur, the diseases are not considered skin diseases, and skin tone is majorly suffered from the ultraviolet rays from the sun. However, dermatologists perform the majority of noninvasive screening tests simply with the naked eye, even though skin illness is a frequent disease for which early detection and classification are essential for patient success and recovery. Due to the ease with which the condition might be missed, this may result in unnecessary diagnostic errors caused by human error. Furthermore, because the symptoms of many common skin diseases share a great deal of similarity, disease classification is challenging [1–4]. Diagnostic procedures need to be precise and timely. Through the application of machine learning algorithms and the utilization of the enormous amount of data present in healthcare facilities and hospitals, artificial intelligence research has recently been utilized in the field of diagnosing skin diseases. The classification of skin diseases using machine learning was the subject of a large number of earlier studies that were compiled in this publication. The researchers used various systems, methods, and algorithms in a collection of prior experiments. Skin disease classification has been accomplished by several methods, with varying degrees of diagnostic precision. Numerous systems have relied on image processing and feature extraction techniques to identify and forecast the type of disease [5, 6]. There are additional techniques created to recognize particular types of skin diseases using clinical characteristics and characteristics discovered by tissue analyses following a skin biopsy of the affected area. In commonly skin diseases are considered conditions and it is affected by our skin the main concepts of skin diseases may be considered as rashes, inflammation, and itchiness or the skin suffering from unwanted facial creams and body creams, thus the skin diseases can be treated by using the various types of treatment and the skin creams and the lotions for the particular skin types. Many skin issues are brought on by the irregular use of skin creams and environmental factors, while some skin conditions may be inherited genetically. In many cases the migration from one to another place causes more and more damage to the skin pattern, thus it affects the skin severely. There are four common skin diseases are found in human beings, mostly these problems are found in all types of skin such as acne; acne is the most common skin disease; the next one is Atopic dermatitis, and this type of skin disease is mostly found the children and also found the early stage of the adults. There are three main reasons are there that the skin tone is damaged, namely, bacteria, viruses, and fungi. These give the most harmful effects on the entire skin tone, Thus, the may form of equipment is used in the medical field, to detect and prevent entire skin diseases [7–9]. The skin treatments are gathered in the following ways including eczema, this eczema is diagnosed in many forms now a day like ointments, lotions, and creams. But the groups of images found in the given dataset are considered as the various forms of the collections, the various skin diseases images are classified are the basis which is in the lack of accuracy in the classification sections and the accuracy of the classification might be handled by the various form of the collections, namely, using deep learning, Artificial intelligence, and the machine learning techniques, thus this paper implements that the hybrid based artificial in the neural approach [10–13]. This section addresses the segmentation and classification approaches employed by various researchers to improve the overall skin lesion categorization in comparison to previous publications. (i) Do not concentrate on organizing multiple image textures. (ii) To do this, color and geometric elements must be taken into account in addition to the texture feature of the patterns, which has not been exploited in this work. (iii) Only Inception v4 was utilized in this segmentation-based classification model for skin lesions to improve performance; it is necessary to look into alternative deep learning models.

This research paper contains Section 2 as a literature review, Section 3 as a proposed methodology, Section 4 as a proposed approach, Section 5 as dataset description, Section 6 as comparative results and analysis, and Section 7 as conclusions and future work.

## 2. Review of Literature

Chen et al. [1] implemented skin diseases recognition based on self-learning and wide data collection through a closed-loop framework, the skin diseases classifications based on the Artificial intelligent technique in the paper the given datasets are experiment checked up in the ways of the LeNet – 5, AlexNet and VGG16. Kawahara et al. [2] implemented the multi-resolution-tract CNN with Hybrid pretrained and skin-lesion trained layers, the multitrained skin classification using the multiple hybrid analysis of the skin texture classification, thus the result of this analysis gives that the enhanced results when compared to the existing technique. Verma et al. [3] presented the Digital Diagnosis of Hand Foot and mouth disease using hybrid Deep Neural Networks, the lightweight, and the hybrid based deep neural perceptrons, the skin diseases are diagnosed by using the Hybrid deep neural network for diagnosis and the datasets are classified by using the MobileNet. Rebouças Filho et al. [4] implemented the Automatic histologically–closer classification of skin lesions, and the feature extraction techniques are handled by using SCM methods from the dataset collection, and the classifications technique are handled by using the Fourier transform and found its accuracy, sensitivity, average, mean correlation, etc., and finally it explains the accuracy classifications of the images. Alsaade et al. [5] implemented the Developing a recognition system for diagnosing melanoma skin lesions using artificial intelligence algorithms for skin disease classification with the perfect accuracy pattern and then the skin diseases are further classified as the various types of techniques. Deepa and Devi [6] implemented the survey on artificial intelligence for medical image classification, the various types of survey used in the classification of the accuracy algorithm, and the detection and prevention of skin diseases earlier. Zhu et al. [7] the Hybrid AI-assistive diagnostic models permit rapid TBS classifications of cervical liquid-based thin-layer cell smears, the accuracy of the classification of the skin diseases is might more crucial nowadays. Hameed et al. [8] implemented an intelligent computer-aided scheme for classifying Multiple skin lesions, the skin diseases are classified by using the Computer-aided Diagnosis System (CAD). Hemanth et al. [9] implemented the enhanced diabetic retinopathy detection and classification approach using a deep convolutional neural network, the new version of the diagnosis of the hybrid approaches in the skin diseases classification. Khan et al. [10] implemented the skin lesions segmentation and multiclass classifications using deep learning features and improved moth flame optimization. Xie et al. [11] implemented the mutual bootstrapping model for automated skin lesion segmentation and classifications. Normally skin cancer classification is one depended on the accuracy of the classification and the segmentation processes, and finally, the results are verified by using the dataset basis. Thapar et al. [12] implemented the novel hybrid deep learning approach for skin lesion segmentation and classification, the classification of skin diseases is classified by using swarm intelligence approaches and the Region of interest (ROI) techniques. Malciu et al. [13] implemented the Artificial Intelligent Based Approaches to Reflectance Confocal Microscopy Image Analysis in Dermatology, the confocal based diagnosis plays a vital role in the form of the classifications of the accuracy in skin diseases. Oliveira et al. [14] implemented the Computational methods for the image segmentation of pigmented skin lesions; skin cancer is considered the most harmful disease nowadays. Rinesh et al. [15] implemented the Investigations on Brain Tumor classifications Using hybrid Machine Learning Algorithms this paper implemented the multicolor representation of the skin in the form of the classifications of the various types of diseases. Połap et al. [16] implemented the intelligent system for Monitoring skin diseases this paper implements that the skin diseases have occurred in the form of melanomas. Hoang et al. [17] implemented the Multiclass skin lesion Classification Using a Novel Lightweight Deep Learning Framework For Smart Healthcare this paper implements the new approach based on the skin lesions classifications. Ismael et al. [18] implemented the Enhanced Deep learning approach for Brain cancer MRI images Classification Using Residual Networks, the classifications of the skin diseases in the form of the various types of skin diseases namely Meningiomas, gliomas, and pituitary tumors. Garnavi et al. [19] implemented the Border detection in dermoscopy images using hybrid thresholding on Optimized color channels, the automatic border detection in the entire datasets, this paper implemented the early collections of the datasets. Chieregatoet et al. [20] implemented the hybrid Machine learning/deep learning COVID-19 severity predictive model from CT images and clinical data this paper proposed the accuracy of the classifications of the images in COVID-19 patients.

## 3. Proposed Methodology

The overview of the proposed approach implies that the basic concepts of the image processing technique should be expressed digitally; mostly the disease classifications are involved only in the form of the various types of the algorithm.

Figure 1 implies that in the overview of the proposed approach, the image processing techniques are involved in the following ways, namely, the given input data sets go through the preprocessing techniques, these techniques are handled by using the median filter in our proposed approach, the preprocessing techniques are helping to remove the noise in the images, the median filter removes the salt and the pepper noise in the given input images.

After the completion of the preprocessing technique, the segmentation process has been handled by reducing the dimensionality space in the entire image thus helping to smoothen and sharpen the edges in the entire image.

After the completion of the segmentation process, the feature extraction process has been taking place, the feature extraction in the entire image processing is considered as the dimensional reduction process, thus the entire dataset individual images are broken up into more manageable groups; in our paper, it is implemented that the given collections for skin diseases are extracted by using the Structural Co-Occurrence matrixes.

This feature extraction plays a vital role in image processing since the better quality the dimensional quality reduction in the entire network system provides enhanced accuracy results in the image classifications.

Our proposed approach provides an enhanced Convolutional Neural Network for the classification of the whole scale images. And, finally, our proposed paper compares with the existing approach in the entire image processing system [21–31].

## 4. Proposed Approach

The proposed implements our proposed technique for the skin disease classifications. The preprocessing filter helps to remove the noise in the entire image, thus it provides a better quality of the image to the segmentation process, and the segmentation process is slightly the same as the feature extraction process; the segmentation process handles that the division or the region of the whole images in the entire network process.

The feature extraction techniques in our proposed methods show that the more valuation results in the entire network, the structural Co-Occurrence is one of the major techniques that provide enhanced accuracy in the entire results in the image processing.

The combination of the feature extraction In SCM and the classification in ECNN shows better accuracy when compared to the existing techniques.

Figure 2 implements the proposed approach for the skin diseases classification, and our proposed method implements the median filter for the preprocessing technique, the preprocessing filter is one the most crucial technique in the image processing system.

### 4.1. Preprocessing

The preprocessing in the image processing helps to remove the noise in the entire image processing technique, and the main function of the image processing technique is to reduce the noise in the image by adding many types of filters, and then the RGB images are converted into the greyscale images, In our paper implements that the median filter for removing the noise in the image. The preprocessing for each image can be gathered by using the following five steps, namely, Image resizing, Transformation to the greyscale images, Noise Removal, segmentation masks, and contrast adjustment. The individual specialty of the median filter is removing the noise in the image by adding salt and pepper to the entire image. The Gaussian and the median filter are considered as the opposite complex filter thus the median filter acts as the intermediate and nonlinear filter in the image processing; it provides the normalization in the given datasets. The Gaussian filer is considered the linear filter in the image processing system.

(1) $$\begin{array}{c} \text{Median value}=\frac{\left(n+1\right)}{2}. \end{array}$$

Equation (1) implies that the median value of the entire network, thus the median filter in the images processing techniques takes place in the two types, namely, maximum filter and the minimum filter; the maximum filter is considered as the high pixel rate of the filter and the minimum filter are considered as the low pixel rate of the filter [32].

### 4.2. Structural Co-Occurrence Matrix

The feature extraction techniques are nothing but the given input images are split up into more manageable groups, and there are many techniques involved in the form of the feature extraction in the skin diseases classifications, namely, GLCM and the LBP techniques are expressed in the [4]. The Structure Co-Occurrence Matrix is of a similar technique; the SCM helps to identify the structure in the entire image, and thus it produces that ensures better accuracy of the feature extraction.

Figure 3 represents the generic Structural Co-Occurrence model in the image processing; the SCM uses the both original image and the filtered images, and the original images are compared with the filtered images [4].

Thus the result of the SCM In the image processing provides better accuracy in the field of image processing. And, the final result gives the input for the classification techniques [4].

### 4.3. Enhanced Convolutional Neural Network

The CNN normally provides better image classifications and also provides better accuracy in the entire image processing techniques; normally, the Convolutional Neural Network provides the three basic functions in the image processing namely max-pooling, fully connected layer, and convolution.

Figure 4 represents the Enhanced Convolutional Neural Network in the image processing; after the completion of the feature Extracting images are given as the input for the classification approaches, thus the convoluting layer takes place through the input images without having noise, since the convolutional layer is inbuilt having the denoising function, thus the completing process of the given datasets gives the input of the Max-pooling function. The main function of the max-pooling reduces the overfitting in the entire images, and the overfitting is considered as the major challenge in the image processing technique.

Specificity: A test's capacity to appropriately identify those who do not have the disease.

True positive: the individual has the disease and the test results are positive; true negative: the individual does not have the disease and the test results are negative.

Index: the Index collects, organises, distils, and visualises artificial intelligence data. We provide policymakers, scholars, journalists, executives, and the general public with unbiased, rigorously validated, and globally sourced data to help them gain a better grasp of the difficult field.

Accuracy: it displays the model's overall accuracy, which is the percentage of total samples correctly identified by the classifier.

(2) $$\begin{array}{c} \text{specificity }=\frac{\text{True negative}}{\text{True negative}+\text{False positive}},\\ \text{Sensitivity}=\frac{\text{True positive}}{\text{True positive}+\text{False negative}},\\ \text{Index}=\text{spec}+\text{sensitivity},\\ \text{Accuracy}=\frac{\text{TP}+\text{TN}}{\text{FP}+\text{FN}+\text{TP}+\text{TN}}. \end{array}$$

## 5. Dataset

There are 3100 Dermoscopy images collected from the PH2 and the ISIC datasets; except for the PH2 datasets, all the datasets are the resizing images, and it has different types of images, and the final results are based on the accuracy results in the form of the melanoma and the nonmelanoma skin diseases classifications.

## 6. Comparison Analysis and Results

According to the Research, melanoma is one of the most common skin diseases all over the world, many researchers are involved to detect and prevent this type of disease but the whole set of data collection provides that the failure results in the accuracy for the classifications of the given datasets, our paper compares that the existing approaches like fast Fourier Transform with the SCM feature extraction and the support vector machine with SCM; the CNN with SCM and the KNN with the SCM, thus our paper implements that the enhanced output compares with the entire results.

Figure 5 implements the comparison results for our proposed approach.

## 7. Conclusion and Future Work

This paper implements that the Structural Co-Occurrence matrices for feature extraction in the skin diseases classification and the preprocessing techniques are handled by using the Median filter, this filter helps to remove the salt and pepper noise in the image processing; thus, it enhances the quality of the images, and normally, the skin diseases are considered as the risk factor in all over the world.

Many researchers are involved to detect and prevent diseases earlier, thus we found this new approach many existing approaches are involved in the classification of the accuracy results in the entire network, and the comparison of our approach provides less amount of accuracy. The simulation results are provided based on the parameters such as accuracy. Our proposed approach provides 97% of the classification of the accuracy results while other existing model such as FFT + SCM gives 80%, SVM + SCM gives 83%, KNN + SCM gives 85%, and SCM + CNN gives 82%.

Future work is dependent on the increased support vector machine's accuracy in classifying skin illnesses, and SCM is used to manage the feature extraction technique.

## Figures and Tables

**Figure 1:** Overview of proposed approach.

**Figure 2:** Proposed approaches.

**Figure 3:** SCM model.

**Figure 4:** Enhanced Convolutional Neural Network. Sensitivity: A test's capacity to correctly identify patients with a condition.

**Figure 5:** Results.

## Data Availability

The datasets used and/or analyzed during the current study are available from the corresponding author on reasonable request.
